The article "Promoting Regional Economic Transformation Forecast Based on Intelligent Computing Technology" was retracted in 2023. Reasons: unreliable results or conclusions; concerns about the data; concerns about the results or conclusions; concerns about the peer review.

# Promoting Regional Economic Transformation Forecast Based on Intelligent Computing Technology

**DOI:** 10.1155/2022/1835376

**Published:** 2022-03-04

**Authors:** Hongbiao Cai

**Affiliations:** Finance Department, Guangzhou Panyu Polytechnic, Guangzhou, Guangdong 511483, China

## Abstract

The core of the value of artificial intelligence is to integrate with the real economy and become more dependent on local industries. In the entire artificial intelligence + industry development process, many new changes have appeared. This article mainly studies how to promote regional economy based on smart technology. In the context of rapid economic development, the significance of artificial intelligence and the necessity of regional economic transformation are put forward. The model has designed the national science and technology mechanism framework from the four directions of technology guidance, technology service, technology innovation, and technology balance; following the cultivating ideas from products to innovative industries to innovative intelligent environments, due to the low income elasticity of product demand, technological innovation is mainly based on the dissemination of emerging technologies outside the industry and the lack of coordination between companies under the fiercely competitive market structure; the focus is on promoting the continuous improvement of labor productivity. The experimental results prove that the emerging technology industries of enterprises can promote economic transformation in the era of artificial intelligence, provide a reference for better optimization of industrial innovation and development, and provide methodological support for the government to establish sound emerging technology business models and optimized management methods.

## 1. Introduction

With the continuous development of computer network technology, artificial intelligence has become a product of technology in the new era. At present, there are many artificial intelligence in life, such as smart TVs, smart phones, and so on, which bring convenience and speed to people's lives. It can be seen that artificial intelligence, a modern technology, has an important impact on people's lives. In artificial intelligence, the application of computer network technology plays an important role. The two influence each other and gradually achieve better development. However, the technical equipment of China's traditional manufacturing industry is relatively backward in general, and the penetration rate of intelligence in traditional manufacturing is low. Traditional manufacturing is still under pressure to adjust structure, reduce production capacity, reduce costs, and increase efficiency, all of which make traditional manufacturing intelligent. Upgrading brings great difficulty.

The article "Promoting Regional Economic Transformation Forecast Based on Intelligent Computing Technology" was retracted in 2023. Reasons: unreliable results or conclusions; concerns about the data; concerns about the results or conclusions; concerns about the peer review.

Artificial intelligence is a modern advanced technological productivity. The application of artificial intelligence technology has brought profound changes in production methods and lifestyles, as well as further liberation of the labor force [1, 2]. The artificial intelligence industry will drive the development of the intelligent economy and will also become a new economic growth point in China in the future. Artificial intelligence technology will become a powerful engine for China's national economic and social development [3, 4]. The artificial intelligence industry will promote the real economy to move towards equipment intelligence, structural optimization, and industrial transformation and quality improvement. At the same time, the evaluation index system of emerging technologies affects traditional industries from the perspective of integrated innovation based on the mechanism of action refines the dimensions of the impact of emerging technologies on traditional industries, which is a further deepening of existing evaluation research and promotes more focused and targeted evaluation analysis. It enriches the perspective of the evaluation research on the impact of emerging technologies on traditional industries.

Foreign research related to financial support to promote economic growth mainly focuses on the relationship between financial growth and economic growth, and considerable progress has been made. Foreign countries use emerging technologies to strengthen the real economy as an important strategic measure and actively promote comprehensive reform and innovation from manufacturers to innovative systems, from business structures to organizational forms, and from development concepts to business models. Goel believes that traditional industries are still playing an important role in promoting the development of new technology industries [5]. Wright proposed that traditional industries can promote and cultivate emerging industries [6]. Arencibia-Jorge et al. use the benign interaction between traditional industries and emerging industries to achieve “two-wheel drive,” which is the key to promoting China's economic growth and ensuring sustainable economic development [7].

In terms of domestic industrial structure, due to the modern technological revolution and the rapid growth of productivity, the industrial structure has gradually moved towards modernization. However, traditional industries use primitive production methods for production; that is, they rely on traditional production technologies, and primitive production technologies particularly rely on directly available resources for production, and the use of labor and capital is inefficient. The rise of emerging technologies contributes to the rise of emerging technology industries and economic growth. The optimization and upgrading of Bychkova's traditional industries can make full use of external factors to develop emerging industries [8]. Harris uses examples of high-tech applications in traditional industries to prove that there is a mutually beneficial relationship between high-tech industries and traditional industries [9].

The article "Promoting Regional Economic Transformation Forecast Based on Intelligent Computing Technology" was retracted in 2023. Reasons: unreliable results or conclusions; concerns about the data; concerns about the results or conclusions; concerns about the peer review.

This paper conducts a longitudinal comparative analysis of the influence of emerging technologies on traditional manufacturing steel in the country and horizontally compares the results of traditional equipment manufacturing and the steel industry; on the basis of clarifying the degree of influence of emerging technologies on traditional industries from the perspective of integrated innovation, corresponding countermeasures and suggestions are put forward. At the same time, electronic interviews were conducted with 4 experts, and the data obtained from the interviews were processed and analyzed. The penetration level of emerging technologies into traditional industries reached 0.420, and the level of absorption and absorption of emerging technologies by traditional industries reached 0.512. Therefore, emerging technology industries have the ability to promote regional economic transformation and upgrading very effectively.

## 2. Research on the Path of Enterprise's Emerging Technology Industry Promoting Regional Economic Transformation and Upgrading

### 2.1. Internet of Things

Judging from the current situation, the system structure of the Internet of Things is not complete [10, 11]. As we know, the Internet of Things is divided into three layers: perception layer [12], network layer [9], and application layer [10]. Its structural model is shown in Figure 1.

### 2.2. Smart Environment

The smart environment is a very interactive system. The environment must be able to perceive people's behavior or situation and be able to accurately read the behavior or situation so as to make judgments to provide the people with corresponding intelligent services [13–15]. Among them, self-perceived mobility and intelligent recognition technology are hot and difficult points of current research. Human-friendly built-in hardware devices, convenient two-way communication mechanism, and security and reliability are one of the most basic technologies for building a smart environment [16, 17]. Due to the complexity of computing components in the environment, many differentiation issues have also been brought about in the design of system applications. In order to protect the differences in the bottom layer, deletion and merging must be performed at a higher level. Standard service description, registration, and inquiry complete a series of customized automated processes at the top of the call and the call, reflecting the functions of the intelligent environment [18, 19].

The article "Promoting Regional Economic Transformation Forecast Based on Intelligent Computing Technology" was retracted in 2023. Reasons: unreliable results or conclusions; concerns about the data; concerns about the results or conclusions; concerns about the peer review.

Smart environment is a new idea and new technology that people put forward in order to make it more convenient for them to serve themselves. Not only must the technical factors be checked, but also personal, cultural, moral, social, and legal factors must be further checked to create a truly intelligent environment [20]. Therefore, the smart environment includes many related industries, including distributed intelligence and data exchange. Distributed intelligence means that ASON realizes the distributed intelligence of the network, that is, the intelligence of network elements, which is embodied in the realization of network topology discovery, route calculation, automatic link configuration, path management and control, and service protection by relying on network elements and recovery functions. Data exchange refers to the process of establishing a temporary interconnection path for data communication between multiple data terminal devices for any two terminal devices.

#### 2.2.1. Related Technology

Intelligent environment technology is the cornerstone of the knowledge search system created in this article, mainly used to solve the problem of knowledge acquisition and integration. The smart environment is essentially a structured semantic network, stored in the form of graphs. The technical fields related to the smart environment are very extensive [21, 22]. Here, the environment-based computers, technologies related to wireless sensors, and activity recognition technologies are analyzed. These three are key areas in the intelligent environment and are closely related to each other: environment-driven computer environment acquisition, modeling, representation processing, and sensor technology are interrelated and closely related. There are many ways to identify activities, and this article uses a method based on sensor activity. The process of reasoning and recognition activities is the upper and lower processing and combined analysis of the environment [23].

#### 2.2.2. Edge Computing in a Smart Environment

There are usually two ways to create a smart environment: a top-down approach and a bottom-up approach. The top-down construction method is an ontology-based construction method, using highly structured encyclopedias and other sites as data sources, from which the constraints and rules of the ontology are extracted and supplemented in the knowledge base, while the bottom-up construction method is simple [24, 25]. By identifying patterns and formulating rules, and then adding them to the smart environment, the collected data is used to identify entities, attributes, and relationships. Due to the rapid development of the Internet of Things, the popularity of wireless network technology, and the rapid increase in the number of edge network devices, the data generated by advanced devices has not yet been effectively processed. This is mainly reflected in the linear growth of computing power and massive data. The transmission of network edge devices to the central node leads to a sharp increase in network transmission, which leads to network delays. Network acne data includes privacy, and transmission of raw data to host nodes may leak privacy. In edge computing, data requests come from the local area and are (pre)processed locally and then sent to the remote server. Data processing and transmission are bottom-up methods.

The article "Promoting Regional Economic Transformation Forecast Based on Intelligent Computing Technology" was retracted in 2023. Reasons: unreliable results or conclusions; concerns about the data; concerns about the results or conclusions; concerns about the peer review.

#### 2.2.3. Integrated Smart Environment

In view of the fact that most research results are based on specific data sources and specific methods, and the built-in intelligent environment of the discipline exposes limited breadth and depth, the universal intelligent environment of the discipline based on bibliographic information design integrates the advantages of various tools and accurately reveals the development of the discipline status quo and the realization of multimethod verification for specific problems [26, 27]. A variety of visualization construction methods integrate a single relationship with data sources, such as keyword co-word relationship clustering tree diagram analysis to reflect the macro structure of the subject, and multidimensional scale analysis to reflect the macro structure of the subject.

### 2.3. Emerging Technologies Affect the Role of Traditional Industries

#### 2.3.1. The Proliferation of Emerging Technologies

Dissemination of emerging technologies to traditional industries refers to the provision of emerging technologies to potential technology users through certain channels. This proliferation is mainly due to the technological gap between the two parties and the transformative power of traditional industries. At the same time, many external groups are promoting the spreading process, restrictions, and risk factors. It mainly comes from the technological gap between the two sides and the transformation power of traditional industries. At the same time, the diffusion process is affected by many external promotions, constraints, and risk factors. Only when there is a technological gradient between emerging technologies and traditional industries and there are appropriate external conditions to drive them, emerging technologies will diffuse through the market or other intermediaries and transfer to traditional industries, as shown in Figure 2.

The article "Promoting Regional Economic Transformation Forecast Based on Intelligent Computing Technology" was retracted in 2023. Reasons: unreliable results or conclusions; concerns about the data; concerns about the results or conclusions; concerns about the peer review.

#### 2.3.2. Acceptance of Traditional Industries

When emerging technologies are transferred to traditional industries through the former market or other intermediaries, the effective penetration of emerging technologies will depend on the acceptance and recognition of emerging technologies by traditional industries. The main body of technology acceptance in traditional industries is enterprises, and the research process of evaluating the impact of emerging technologies on traditional industries from the perspective of specific acceptance of integrated innovation is as follows: enterprise decision makers conduct market demand analysis in combination with the market environment, and on this basis, according to the enterprise's own resource conditions and technical capabilities, it decides whether to adopt and which appropriate emerging technologies to adopt to transform the enterprise, so as to achieve the improvement of the technical level, as shown in Figure 3.

#### 2.3.3. Integration of Emerging Technologies and Traditional Industries

As the latest technology in the current field, emerging technologies have the characteristics of high penetration. With the penetration of emerging technologies in traditional industries, traditional industries will undergo qualitative changes in terms of technological foundation, product structure or overall industrial structure. These changes will form interactions in the external environment. The specific fusion process is shown in Figure 4.

As shown in Figure 4, after traditional industries accept the entry of emerging industries, traditional enterprises start from five major aspects, including products, process equipment, and management methods. Promote the improvement of the technological level of enterprises and realize the upgrading of traditional industries.

### 2.4. The Relationship between Emerging Technologies and Traditional Industries

The role of integrated innovation is to promote the integration of technological resources and industrial development. The essence of the role of emerging technologies and traditional industries is to accept, integrate, and integrate emerging technologies from traditional industries, thereby promoting the transformation and upgrading of traditional industries. It can be seen that integrated innovation is an important aspect of industrial development [28, 29]. Therefore, this article explores the relationship between emerging technologies and traditional industries from the perspective of integrated innovation. Through the analysis of the tone, stage, and specific impact of emerging technologies affecting the transformation of traditional industries, the specific relationship between emerging technologies affecting traditional industries is discussed from the perspective of integrated innovation, and the theoretical basis of innovation is discussed theoretically.

The article "Promoting Regional Economic Transformation Forecast Based on Intelligent Computing Technology" was retracted in 2023. Reasons: unreliable results or conclusions; concerns about the data; concerns about the results or conclusions; concerns about the peer review.

The impact of emerging technologies on traditional industries is not only the process of technological progress, but also technological and economic activities. On the one hand, the essence of the transformation of traditional industries from emerging technologies is to gradually upgrade the industrial structure through the diffusion and penetration of emerging technologies, thereby realizing the progress of the industrial structure and leading technological progress [30]; on the other hand, emerging technologies have also provided great help to the transformation and upgrading of traditional industries. The factors of production are being stabilized, as well as the existing economic organizations' understanding of emerging technologies and their participants. This process can effectively improve the production technology level of traditional industries, increase production efficiency, improve corporate governance, effectively reduce product quality, effectively reduce resource consumption and environmental pollution, eliminate useless production capacity, and maintain efficient production capacity. Only when emerging technologies gradually penetrate into traditional industries, and traditional industries decide to accept them, can the two achieve integration and integration, and diffusion and absorption are deeply embedded in the integration process. Therefore, from the perspective of integrated innovation, the essence of the process of emerging technologies affecting traditional industries is the optimal allocation and synergistic integration of existing production factors of traditional industries and innovative factors of emerging technologies.

The introduction of emerging technologies will penetrate all aspects of traditional industries and then lead to a series of changes in traditional industries, such as business philosophy, production management, employment, and systems. It is a process of coordination and integration of various themes or elements, reflecting the characteristics of the system. The impact of technology on traditional industries not only involves the application of new technologies and new processes, but also includes enhancing traditional industries' awareness of concepts, management, markets, and technological innovation through technology penetration; marketing is one of them. Basically, according to the market environment, it can play its potential from emerging technologies and the sources of emerging technologies and play a role in traditional industries. The impact of emerging technologies on traditional industries is also in line with the basic laws of market economy; the process of emerging technologies operating in traditional industries is a technological and economic activity. The fundamental purpose of using emerging technologies to operate in traditional industries is to promote the transformation and upgrading of traditional industries and optimize production capacity through structural adjustments, thereby stimulating economic growth. It can be regarded as an investment and development behavior, and it is a feature of high technology. In contrast, the biggest feature of emerging technologies is “Xing,” which means that they are emerging and coming into effect. In other words, the usefulness of emerging technologies usually takes some time. The use of emerging technologies to transform traditional industries will be a long-term process of change. The absorption of emerging technologies by traditional industries will not only be based on the immediate transformation of emerging technologies, but will also make full use of them. The potential energy of emerging technologies is improving and adapting to the industry.

The article "Promoting Regional Economic Transformation Forecast Based on Intelligent Computing Technology" was retracted in 2023. Reasons: unreliable results or conclusions; concerns about the data; concerns about the results or conclusions; concerns about the peer review.

## 3. Experimental Research on the Path of Enterprise's Emerging Technology Industry Promoting Regional Economic Transformation and Upgrading in Intelligent Environment

### 3.1. Test Subject

In this study, four experts who are most interested in innovation theory or industrial development were invited to evaluate indicators at all levels of the integration and integration of emerging technologies and traditional industries. Experts include 2 X University professors and 2 bosses who have successfully transformed design and manufacturing enterprises. The scoring format is completed through electronic interviews. By constructing a questionnaire about the relationship between evaluation indicators of emerging technologies affecting traditional industries from the perspective of comprehensive innovation, it provides a data basis for analytic hierarchy process used to obtain the weight of each indicator.

### 3.2. To Gather Data

According to the expert questionnaire survey, calculate the average value of the expert data, a matrix *X* can be obtained, which needs to meet *a*_*ij*_ > 0, *a*_*ij*_=1/*a*_*ji*_, *a*_*ii*_=1, where *i*, *j* = 1, 2,…, *n*.

(1) $$\begin{array}{c} X=\left[\begin{array}{ccc} a_{11} & \cdots & a_{1n}\\ \vdots & \ddots & \vdots \\ a_{n1} & \cdots & a_{nn} \end{array}\right]. \end{array}$$

The square root method is used to measure the weight of each index. The specific formula is shown as follows:

(2) $$\begin{array}{c} h_{i}=\sqrt[{n}]{\prod_{i=n}^{n}a_{ij}}. \end{array}$$

The weights *w*_*i*_ of the possible indicators are as follows:

(3) $$\begin{array}{c} w_{i}=\frac{h_{i}}{\sum_{i=1}^{n}h_{i}}. \end{array}$$

The calculated indicator weight is only lower than the indicator weight of each standard level. The weight of each indicator in the entire indicator system should be further converted according to the dimensions of the standard level.

The article "Promoting Regional Economic Transformation Forecast Based on Intelligent Computing Technology" was retracted in 2023. Reasons: unreliable results or conclusions; concerns about the data; concerns about the results or conclusions; concerns about the peer review.

### 3.3. Experiment Procedure

#### 3.3.1. Experiment Preparation Stage

By reviewing relevant literature, construct a questionnaire on the relationship between the evaluation indicators of emerging technologies affecting traditional industries so that the volunteers can perform the next step in the trial phase.

#### 3.3.2. Experimental Stage

Interviews were conducted with 4 experts via telephone voice to obtain experimental data. And these data were organized for the next step to calculate the data, and analyze the conclusions of the next step through these results.

#### 3.3.3. End of Experiment

Discuss and analyze the data results obtained in the experimental stage, combine some knowledge theories and horizontally compare the results of traditional equipment manufacturing and steel industry, and put forward corresponding suggestions on the basis of clarifying the impact of emerging technologies on traditional industries from the perspective of integrated innovation countermeasures and suggestions.

### 3.4. Data Processing

By sorting out the scoring tables filled out by 4 experts, 4 judgment matrices for the integration effect of emerging technologies and traditional industries were calculated. The judgment matrix of the second-level index is *u*; the judgment matrix of the third-level index is *u*_1_. Since this paper has a three-level index system, it is necessary to carry out a multilevel fuzzy comprehensive evaluation. That is, the first-level comprehensive evaluation is carried out on the first-level scope, and then the second-level comprehensive evaluation is carried out according to the evaluation results, and so on.

(4) $$\begin{array}{c} u=\left[\begin{array}{ccc} 1 & 0.9 & 3\\ 1 & 1 & 5\\ 0.3 & 0.2 & 1 \end{array}\right],\\ u_{1}=\left[\begin{array}{cc} 1 & 0.78\\ 1/0.78 & 1 \end{array}\right]. \end{array}$$

The statistical data used in this article has a different unit dimension for each index data, so the corresponding calculation cannot be directly performed in the overall evaluation. First of all, index data must be processed without dimension, that is, normalization. The common method of data standardization is usually min-max standardization. This method can evenly distribute the index data to the range [0–1]. The indicators selected in this paper have practical significance and are all positive indicators, so it is more suitable to use this method for dimensionlessization. The calculation formula of this method is shown in

(5) $$\begin{array}{c} x=\frac{x-\min}{\max-\min}. \end{array}$$

The specific formula is as follows:

Large trapezoidal distribution:

(6) $$\begin{array}{c} r\left(x\right)=\frac{x-c}{d-c},\;c<x<d. \end{array}$$

Small trapezoidal distribution:

(7) $$\begin{array}{c} r\left(x\right)=\frac{b-x}{x-a},\;a<x<b. \end{array}$$

For the ideal score value, it can usually be set as the middle value of each interval. This paper divides the evaluation grades into five grades, and the index data after normalization processing all fall in the [0–1] interval.

The article "Promoting Regional Economic Transformation Forecast Based on Intelligent Computing Technology" was retracted in 2023. Reasons: unreliable results or conclusions; concerns about the data; concerns about the results or conclusions; concerns about the peer review.

### 3.5. Clustering Algorithm Based on Intelligent Technology

Clustering originated from data taxonomy, so clustering and classification have a certain connection and similarity, but there is still a certain difference from classification. The clustering algorithm is shown in Figure 5.

As shown in Figure 5, it can be seen that the essence of clustering is not knowing the category or other prior knowledge of each sample in a batch of samples in advance.

#### 3.5.1. Cohesive Hierarchical Clustering Method

Contrary to the split hierarchical clustering method, the agglomerative hierarchical clustering method first treats each object as a class and then aggregates these nodes in turn to form the nodes of the upper level tree until all the nodes are merged into one large category, or until a termination condition is reached, as shown in Figure 6.

As shown in Figure 6, let the random matrix be *W*, and let lim*W*^*m*^ be the primitive random matrix of $W=\lim W^{m}=\left[\begin{array}{cc} c^{\infty } & 0\\ r^{\infty } & 0 \end{array}\right]$; then, the following matrix is a stable random matrix as follows:

(8) $$\begin{array}{c} W=\lim W^{m}=\left[\begin{array}{cc} c^{\infty } & 0\\ r^{\infty } & 0 \end{array}\right]. \end{array}$$

Suppose a set of samples is *a*_*i*_, and the sample has *n* features; then, the sample vector is

(9) $$\begin{array}{c} a_{i}=\left\{a_{1},a_{2},\ldots a_{n}\right\}. \end{array}$$

Taking Euclidean distance as the distance between the sample and the cluster center, the process of minimizing the transition of the clustering process is given by

(10) $$\begin{array}{c} f\left(a,b\right)=\sum_{j=1}^{d}u_{ij}. \end{array}$$

Finding the smallest point (*a*, *b*) in formula (10), Euclidean distance is

(11) $$\begin{array}{c} u_{i}=\frac{\sum_{j=1}^{d}u_{ij}*a^{i}}{\sum_{j=1}^{d}u_{ij}}. \end{array}$$

The cluster center *u*_*ij*_ of the class is

(12) $$\begin{array}{c} u_{ij}=\frac{1}{\sum_{i=1}^{c}{\left(2/d_{ij}\right)}^{2}}*{\left(\frac{2}{d_{ij}}\right)}^{2}. \end{array}$$

The clustering feature tree is a highly balanced tree that is used to store the feature information of the cluster, and it occupies a small space and can be stored in the memory, thereby improving the clustering speed and scalability of the algorithm on large data sets, as shown in Figure 7.

The article "Promoting Regional Economic Transformation Forecast Based on Intelligent Computing Technology" was retracted in 2023. Reasons: unreliable results or conclusions; concerns about the data; concerns about the results or conclusions; concerns about the peer review.

As shown in Figure 7, the algorithm is mainly divided into two stages: the first stage uses hierarchical clustering; after meeting certain requirements, other division methods are used for macro-clustering processing.

It is assumed that the current optimal position of the entire fish school is to speed up the search speed of the algorithm. In the rear-end collision operation, the global optimal position at this moment is used to replace the optimal position of the individual fish neighborhood.

(13) $$\begin{array}{c} a_{i}=a_{i}+\text{rand}\left(\text{step}\right)\frac{a_{g\text{best}}-a_{i}}{\left\|a_{g\text{best}}-a_{i}\right\|}, \end{array}$$

where *a*_*g*best_ represents the optimal position of the entire school of fish.

Then, the access sequence length weight can be calculated as

(14) lwi=1−leni−lenlen−maxlen.

Taking *lw*_*i*_ as a penalty factor means that the closer the length of the access sequence is to the length of the average access sequence, the larger the value of the factor is, and vice versa, the smaller the value of the factor is.

### 3.6. Data Preprocessing Based on Smart Technology

Preprocessing is the most critical link to ensure that the correct and useful patterns can be discovered efficiently and quickly. The function of this module is to process log files in different types of formats and convert them into data in a unified format that the system can handle; at the same time, it is necessary to complete the cleanup of log data and the identification of access sequences, as shown in Figure 8.

As shown in Figure 8, in this general model of intelligent computing, the key issue is to study how simple individuals can form high-level systems with complex intelligent behaviors under the guidance of simple interaction rules, as shown in Figure 9.

As shown in Figure 9, a complex computing task is completed by a large number of nonsimultaneous computing behaviors of computing units; all the characteristics of the units performing these tasks 3 are unknown to other units and even the system itself; the behavior of a large number of units is determined based on the fact that they are based on incomplete knowledge of the system and delayed or even contradictory information.

The article "Promoting Regional Economic Transformation Forecast Based on Intelligent Computing Technology" was retracted in 2023. Reasons: unreliable results or conclusions; concerns about the data; concerns about the results or conclusions; concerns about the peer review.

## 4. An Experimental Analysis of the Path of Enterprises' Emerging Technology Industry in Promoting Regional Economic Transformation and Upgrading in an Intelligent Environment

### 4.1. Analysis of the Weight of Emerging Technology Industry in Promoting the Transformation and Upgrading of Regional Economy

According to the formula of calculating the index weight by the analytic hierarchy process, the weight of the first-level index can be obtained, and the reliability CR = 0.022 is less than 0.05, so the weight distribution meets the requirements. Furthermore, the weight of each secondary indicator can be obtained. The reliability CR = 0.013 is also less than 0.05, and the weight distribution also meets the requirements. Therefore, the weight of each three-level indicator can be obtained and converted into the overall indicator weight. The impact of emerging technologies on traditional industries is shown. The total weight of the impact evaluation is shown in Table 1.

It can be seen from Table 1 that the data obtained from the experiment is processed and analyzed. The impact level of emerging technologies on traditional industries reaches 0.420, and the external support level is only 0.114, which can make the traditional industries absorb emerging technologies as high as 0.512, so the emerging technology industries are promoted. The transformation and upgrading of the regional economy has been very effective.

### 4.2. Comparative Analysis of Indicators within and between Industries over the Years

#### 4.2.1. Comparative Analysis within the Industry

Figure 10 shows the impact level of emerging technologies on the traditional equipment manufacturing industry and the steel industry, the level of digestion and absorption of traditional industries, the level of external support, and the effect of integration from 2015 to 2020. On this basis, corresponding countermeasures and suggestions are put forward, as shown in Figure 10.

It can be seen from Figure 5 that, as time goes by, the integration and integration of emerging technologies and traditional equipment manufacturing has continued to increase. First, the penetration level of emerging technologies in the traditional equipment industry is on the rise, reaching the highest level by 2019. The main reason is that the traditional equipment industry has continuously strengthened the introduction and absorption of new technologies in recent years. Under the influence of new technologies, there is a steady-increase investment in existing technology transformation and R&D.

The article "Promoting Regional Economic Transformation Forecast Based on Intelligent Computing Technology" was retracted in 2023. Reasons: unreliable results or conclusions; concerns about the data; concerns about the results or conclusions; concerns about the peer review.

#### 4.2.2. Comparative Analysis between Industries

Through internal comparison, we can discover various reasons or factors of how emerging technologies in industry effectively affect traditional industries. In order to further analyze the common factors of the impact of emerging technologies on different traditional industries, it is also necessary to conduct a horizontal comparison and analysis of the evaluation results of different industries to find common points and make more comprehensive recommendations, as shown in Figure 11.

It can be seen from Figure 6 that from the perspective of the penetration level of emerging technologies in the traditional equipment industry and the steel industry, the introduction of emerging technologies in the steel industry was earlier and led the traditional equipment industry before 2015. Since 2015, the traditional equipment industry has been stable. However, the steel industry has experienced a shocking decline. The steel industry is gradually surpassing the traditional equipment manufacturing industry. The traditional equipment industry is more receptive to emerging technologies, and the ability to raise funds from all aspects is becoming stronger.

After a comprehensive analysis of the results, we found that the evaluation results of the integration and fusion of traditional equipment manufacturing and steel industry with emerging technologies are all on the rise, which shows that the integration and integration of emerging technologies and traditional industries is increasing. The bad gradually turned into better or even very good. This also reflects from the side that my country's traditional equipment manufacturing industry and steel industry have effectively used emerging technologies to promote the gradual innovation and development of the industry.

### 4.3. Analysis of Hausman Test Method

#### 4.3.1. LM Detection Analysis

This document uses the least squares method to estimate the usual table data model, which does not consider the spatial correlation, and then verifies the spatial correlation of the model residuals. The main test methods are Lmsar, Lmerr, R-Lmsar, R-Lmerr, and so on. If Lmsar is better than Lmerr, and R-Lmsar is important, and Rt-Lmerr is not important, the spatial delay table data model is better than the spatial error table data model. See Figure 12.

According to the results of the LM test, determine whether the spatial measurement model should use fixed effects or random effects. The result of LM test passed the significance test of 0.005. Therefore, this article will deal with fixed-effect time models, fixed-space models, and dual fixed-space and time models. The estimated results are shown in Table 2.

The article "Promoting Regional Economic Transformation Forecast Based on Intelligent Computing Technology" was retracted in 2023. Reasons: unreliable results or conclusions; concerns about the data; concerns about the results or conclusions; concerns about the peer review.

Combining the results of Figure 7 with the results of Table 2, it can be seen that the coefficient of determination and the adjusted coefficient of determination of the spatial panel regression results are significantly better than the ordinary panel regression results, which indicates that the spatial table data model is effective in affecting coupling and coupling. Factors have stronger explanatory power. Commonly used tabular data model analysis industry and traditional industry.

#### 4.3.2. Unit Root Risk Analysis

The test methods are Lmsar, Lmerr, R-Lmsar, and R-Lmerr through natural logarithmic transformation to obtain their ADF statistic values at 1% critical value, 5% critical value, and 10% critical value and perform a unit root test on it as shown in Figure 13.

It is easier to obtain ADF test statistics and the corresponding critical values of Lmsar and Lmerr sequences. When the significance level is 1%, the value of statistical control is greater than the critical value, so the Lmsar and Lmerr sequences are both nonstatic sequences, and both are 1. The level differences of R-Lmsar and R-Lmerr tests are both smaller than the corresponding critical value. It can be seen that R-Lmsar and R-Lmerr are stable. Therefore, it can be determined that the root unit roots of Lmsar and Lmerr are a series of first-order integer monosyllables, satisfying the hypothesis of coupling test.

## 5. Conclusion

This article mainly expounds the concept of intelligent computing technology and regional economic transformation. In the method part, it proposes a clustering algorithm based on artificial intelligence technology and uses the clustering algorithm to analyze how to play its role in promoting regional economic transformation. As an important subject of development economics, regional economy has strict connotations: how to effectively use human, material, and financial resources to achieve optimal development in a geographical area with basically similar natural environment and humanistic conditions. It is indispensable to constantly update. The research results show that the intelligent computing technology industry has a strong impact on the domestic regional economy in both the short term and the long term, and cities, especially megacities, have further improved the production automation and production. The degree of intelligence, and at the same time, more and more capital replacement labor, has promoted the increase in total factor productivity and promoted the high-quality development of the regional economy; the vigorous development of the domestic regional economy has promoted the sound development of intelligent computing technology, but the intelligent computing technology has further expanded regional economic development differences. Finally, in order to promote intelligent computing technology to promote the high-quality development of regional economy, it is proposed to further create a good innovation environment for the development of intelligent computing technology.

The article "Promoting Regional Economic Transformation Forecast Based on Intelligent Computing Technology" was retracted in 2023. Reasons: unreliable results or conclusions; concerns about the data; concerns about the results or conclusions; concerns about the peer review.

The influence of the integration of emerging technologies with China's traditional arms industry and steel industry is steadily increasing every year. This shows that from the perspective of integrated innovation, the impact of emerging technologies on Chinese traditional industries is increasing every year, which is consistent with the emergence of emerging technologies. Traditional industries have relatively low direct consumption rates and overall consumption rates for strategic emerging industries, while consumption rates for new energy, new materials and latest equipment industries are relatively high. For the new generation of information technology, the consumption rate of organic, energy-saving, and environmentally friendly, and the new energy automobile industry is very low.

## Figures and Tables

**Figure 1:** Internet of Things system composition diagram.

**Figure 2:** Flowchart of the diffusion of emerging technologies to traditional industries.

**Figure 3:** Flowchart of traditional industries' acceptance of new and new technologies.

**Figure 4:** Flowchart of integration of emerging technologies and traditional industries.

**Figure 5:** Clustering algorithm.

**Figure 6:** Agglomerative hierarchical clustering method.

**Figure 7:** Clustering feature tree.

**Figure 8:** Data preprocessing.

**Figure 9:** Intelligent computing theoretical model framework.

**Figure 10:** Comparative analysis of various indicators of traditional equipment manufacturing.

**Figure 11:** Comparison of penetration levels of emerging technologies in the two major industries.

**Figure 12:** LM test results.

**Figure 13:** ADF inspection result graph's approximate value.

**Table 1:** Weight distribution of evaluation index system.

Level indicator	Secondary indicators	Level-three indicators	Weights
The effect of the integration of emerging technologies and traditional industries	The level of influence of emerging technologies on traditional 0.420	Emerging technology introduction expenditure 0.132	0.372
		Technology and absorption expenditure 0.113	0.238
		Technical transformation expenditure 0.063	0.136
	Traditional industries' digestion level of emerging technologies 0.512	New product sales revenue 0.217	0.367
		The total profit 0.057	0.112
		Number of new product development projects 0.118	0.210
	External support level 0.125	Funds for scientific and technological activities 0.050	0.429
		Tax deduction for technology development 0.057	0.547

The article "Promoting Regional Economic Transformation Forecast Based on Intelligent Computing Technology" was retracted in 2023. Reasons: unreliable results or conclusions; concerns about the data; concerns about the results or conclusions; concerns about the peer review.

**Table 2:** The results of the LM test.

Variable	Fixed effect		
	Fixed time	Space fixed	Fixed time and space
Lmsar	0.187	0.176	0.148
Lmerr	3.122	0.469	0.332
R-Lmsar	0.134	0.114	0.085
R-Lmerr	3.117	0.452	0.324

## Data Availability

No data were used to support this study.
